# Identification of Potential Key Biomarkers of Atrial Fibrillation and Their Correlation with Immune Infiltration in Atrial Tissue

This article has been retracted.

**DOI:** 10.1155/2022/4029840

**Published:** 2022-03-01

**Authors:** Jie Liu, Meilin Liu, Xiahuan Chen

**Affiliations:** Department of Geriatrics, Peking University First Hospital, Beijing, China 100034

## Abstract

**Objective:**

To identify potential key biomarkers and characterize immune infiltration in atrial tissue of patients with atrial fibrillation (AF) through bioinformatics analysis.

**Methods:**

Differentially expressed genes (DEGs) were identified by the LIMMA package in Bioconductor, and functional and pathway enrichment analyses were undertaken using GO and KEGG. The LASSO logistic regression and BORUTA algorithm were employed to screen for potential novel key markers of AF from all DEGs. Gene set variation analysis was also performed. Single-sample gene set enrichment analysis was employed to quantify the infiltration levels for each immune cell type, and the correlation between hub genes and infiltrating immune cells was analyzed.

**Results:**

A total of 52 DEGs were identified, including of 26 downregulated DEGs and 26 upregulated DEGs. DEGs were primarily enriched in the Major Histocompatibility Complex class II protein complex, glucose homeostasis, protein tetramerization, regulation of synapse organization, cytokine activity, heart morphogenesis, and blood circulation. Three downregulated genes and three upregulated genes were screened by LASSO logistic regression and the BORUTA algorithm. Finally, immune infiltration analysis indicated that the atrial tissue of AF patients contained significant infiltration of APC_co_inhibition, Mast_cell, neutrophils, pDCs, T_cell_costimulation, and Th1_cells compared with paired sinus rhythm (SR) atrial tissue, and the three downregulated genes were negatively correlated with the six kinds of immune cells mentioned above.

**Conclusion:**

The hub genes identified in this study and the differences in immune infiltration of atrial tissue observed between AF and SR tissue might help to characterize the occurrence and progression of AF.

## 1. Introduction

Atrial fibrillation (AF) is a type of supraventricular tachyarrhythmia that is characterized by rapid and disordered atrial electrical activity [1]. AF has been determined to affect up to 1% of the general population worldwide, and its prevalence increases exponentially with age, possibly reaching 8% in the elderly population (age > 80 years) [2]. AF has a notable correlation with the occurrence of heart failure and myocardial infarction and stroke, which increases the economic burden on patients' families and society [3]. Therefore, it is highly important to identify the cause of AF and devise an effective treatment method. However, no consensus has been reached concerning the exact etiology and pathological changes involved in AF. Previous studies have shown that the etiology of AF is multifactorial, including both genetic and nongenetic factors. Nongenetic factors that are considered to contribute to the development of AF include age, gender, smoking, obesity, diabetes, hypertension, ischemic heart disease, and valvular heart disease [4]. Several recent studies have employed genome-wide association studies (GWASs) to identify over 100 genetic loci associated with AF, including PITX2, TBX5, PRRX1, and ZFHX3 [5–7]. These genetic factors serve to establish electrophysiological substrates that determine individual vulnerability to AF occurrence and maintenance [8]. However, to date, few studies have investigated the molecular mechanism underlying the pathology of AF.

With the rapid development of science and technology, bioinformatics has provided a powerful strategy for screening molecular markers to elucidate molecular mechanisms [9]. Gene chips have been employed to achieve high-efficiency and large-scale acquisition of biological information to produce comprehensive overviews of genetic networks, and the expression profile data regarding diseases can be obtained on a large scale [10]. In the present study, we first downloaded the microarray dataset for AF from the Gene Expression Omnibus (GEO), and we subsequently analyzed the gene chip by using bioinformatic tools. The immune infiltration in the atrial tissue of AF and sinus rhythm (SR) patients was analyzed by performing single-sample gene set enrichment analysis (ssGSEA). Our objectives were to screen the differentially expressed genes (DEGs) as potential novel biomarkers, identify their correlations with immune infiltration in atrial tissue, and explore the molecular mechanism underlying the pathology of AF; these aims are of considerable research importance.

## 2. Materials and Methods

### 2.1. Microarray Data of Date Preprocessing

The datasets of gene expression profiles in human tissue from left atrial appendage (LAA) with the sequence numbers of GSE14975 (*n* = 10; AF 5; SR 5) and GSE79768 (*n* = 26; AF 14; SR 12) were downloaded from the Gene Expression Omnibus (GEO) database affiliated to the National Center for Biotechnology Information (NCBI) (https://www.ncbi.nlm.nih.gov/geo/) and analyzed on the GPL570 platform ([HG-U133_Plus_2] Affymetrix Human Genome U133 Plus 2.0 Array). Subsequently, the *κ*-nearest neighbor (*κ*NN) method was employed to supplement missing data, and the “*sva*” package (3.32.1 version) (https://bioconductor.org/packages/release/bioc/html/sva.html) was utilized to merge the GSE14975 and GSE79768 gene expression matrices and remove the interbatch differences [11, 12]. Principal component analysis (PCA) was subsequently conducted to view data structures. The flowchart diagram of the materials and methods is presented in Figure 1.

### 2.2. Identification of DEGs

The raw microarray data of the dataset were processed with the “limma” package [13] of the R language to identify the DEGs between AF patients and people with SR. DEGs were identified using a *p* value < 0.05 and ∣Fold Change (FC) | ≥1.5 as criteria; genes were considered to be upregulated if the FC was ≥1.5 and downregulated if the FC was ≤-1.5. The RStudio (v1.2.5019) and library ggplot2 package were employed to create the volcano plot. Finally, the “pheatmap” package [14] of R software was utilized to generate heatmaps.

### 2.3. GO and KEGG Pathway Enrichment Analysis

To obtain biological functions and signaling pathways involved in the development of AF, metascape databases (http://www.metascape.org/) were utilized to annotate and visualize specific genes for Gene Ontology (GO) and Kyoto Encyclopedia of Genes and Genomes (KEGG) pathway enrichment analysis using the clusterProfiler package in Bioconductor. GO analysis is a commonly employed approach for annotating genes and analyzing their biological processes [15]. The KEGG pathway database contains advanced functional data on networks of molecules or genes [16]. Min overlap ≥ 3 and *p* values < 0.05 were considered to be significant.

### 2.4. LASSO Logistic Regression and BORUTA Algorithm

In this study, we employed least absolute shrinkage and selection operator (LASSO) logistic regression and the BORUTA machine learning algorithm to select the diagnostic key markers for AF. The LASSO algorithm was applied with the “glmnet” package [17]. Moreover, BORUTA, a feature selection algorithm, randomly disrupted the order of each real feature, evaluated the importance of each feature, and iteratively removed features with low correlation to determine the best variable. To further identify the diagnostic value of these biomarkers for AF, a total of 500 trees were constructed using the “BORUTA” package for feature selection.

### 2.5. ROC Curve Analysis and Circos Analysis

To confirm the reliability and validity of these hub genes, we utilized other AF cohorts from the GEO database, and normalized matrix files were downloaded. Finally, we selected the GSE41177 dataset (*n* = 38; AF 32; SR 6; GPL570 platform) to validate the results. The *pROC* package was employed to calculate the area under the curve (AUC) of the receiver-operating characteristic (ROC) curve in the test set [18]. Finally, Circos analysis was utilized to visualize the relationships among these diagnostic genes.

### 2.6. Gene Set Variation Analysis (GSVA)

GSVA is a nonparametric and unsupervised algorithm for evaluating the enrichment of transcriptome gene sets by synthetically scoring the gene set of interest. The gene level change was transformed into the pathway level change to determine the biological function of the sample. We employed the GSVA_1.30.0 package in R to evaluate the *t* score and assign pathway activity conditions.

### 2.7. Immune Infiltration by ssGSEA Analysis and Correlation Analysis

We quantified the infiltration levels for each immune cell type by single-sample gene set enrichment analysis (ssGSEA) in the R package GSVA [19]. The ssGSEA utilized the scoring result for individual samples. Next, Spearman correlation between the novel key gene expressions and immune cells was performed by using the “*ggstatsplot*” package (https://github.com/IndrajeetPatil/ggstatsplot).

## 3. Results

### 3.1. Data Preprocessing and Identification of DEGs

We removed the interbatch difference from the gene expression matrix after combining the GSE14975 and GSE79768 datasets, standardized the merged gene expression matrix, and presented the results in a two-dimensional PCA cluster diagram before and after normalization (Figures 2(a) and 2(b)). Our data showed that the clustering of the two groups of samples was more obvious after normalization, indicating that the sample source was reliable. Next, the gene expression matrix was analyzed by using R software, and a total of 52 DEGs were detected, consisting of 26 downregulated DEGs and 26 upregulated DEGs. Also, the heatmap and volcano plot of all DEGs are presented in Figures 2(c) and 2(d), respectively.

### 3.2. GO and KEGG Pathway Enrichment Analysis

GO and KEGG pathway enrichment analysis indicated that these DEGs were significantly enriched in the Major Histocompatibility Complex (MHC) class II protein complex, glucose homeostasis, protein tetramerization, regulation of synapse organization, cytokine activity, heart morphogenesis, and blood circulation (Figure 3(a)). Moreover, we observed that the seven pathways were significantly associated with one another (Figure 3(b)).

### 3.3. Screening and Verification of Novel Marker Genes

We employed LASSO logistic regression and the BORUTA algorithm to perform the next screening of the above mentioned 52 DEGs. The key gene markers obtained by the two algorithms overlapped, and six key genes, consisting of three downregulated genes (CHRNA5, LOC150051, and PP12719) and three upregulated genes (DHRS9, LOC101928304, and RYR1), were screened as novel gene markers for AF (Figures 4(a)–4(d)). To further identify the diagnostic efficacy of these six genes, we validated them with the GSE41177 dataset as the validation set.  Figure 5 shows that the expression levels of these hub genes were clearly different between AF patients and SR controls. Next, the six genes were singly fitted into one variable, and the diagnostic efficiency was determined to be 1 in the test set. ROC analysis showed that the AUC of every key gene model had better predictive power for the occurrence of AF, indicating that these six genes had strong diagnostic value (Figure 6). Finally, Circos analysis showed that CHRNA5 and PP12719 were positively correlated with LOC150051 and that DHRS9 was positively correlated with LOC101928304, while CHRNA5 and PP12719 were negatively correlated with DHRS9 and LOC101928304, respectively (Figure 7).

### 3.4. Biological Function of the Key Genes

To determine the biological function of the novel marker genes, GSVA analysis was employed to investigate the effects of the six genes at the pathway level. The data showed that CHRNA5, DHRS9, LOC101928304, LOC150051, PP12719, and RYR1 were involved in the positive and negative regulation of multiple pathways (Figure 8).

### 3.5. Immune Infiltration Analyses

Using ssGSEA, we first analyzed the difference in immune infiltration between the atrial tissue of the AF group and that of the SR group. The violin plot revealed that the atrial tissue of AF patients generally contained significant infiltration of APC_co_inhibition, Mast_cell, neutrophils, pDCs, T_cell_costimulation, and Th1_cells compared with paired SR atrial tissue (Figure 9(a)). Furthermore, we calculated the correlation between immune infiltration and the novel key genes in the outcome model. Spearman correlation analysis showed that CHRNA5, LOC150051, and PP12719 were negatively correlated with the six kinds of immune cells mentioned above (Figure 9(b)).

## 4. Discussion

At present, numerous studies have demonstrated that the occurrence and maintenance of AF are complex biological processes and represent the ultimate manifestations of numerous cardiovascular and cerebrovascular complications and events. However, the exact etiology and molecular pathological basis of AF have not been elucidated to date. Although the clinical risk factors for this disease are complex and may be aging-related, AF is considered to be heritable. The Framingham Heart Study found that 30% of participants with AF had at least one parent with AF, and individuals with at least one parent suffering from AF exhibited an approximately 40% increased risk of developing AF after adjusting for age, sex, blood pressure, diabetes, and clinically overt heart disease [20]. Moreover, Ellinor and colleagues reported that lone AF significantly increased the risk of AF in family members, and a family history of AF was observed in 38% of patients with lone AF [21]. These results indicate a potential role for genetic variations in the pathophysiology of AF. In recent years, the rapid development of bioinformatic methods has facilitated the study of genomic mapping and epigenomics, contributing to more in-depth identification and annotation of important functional regulatory elements in disease or morphological development and outlining hub gene regulatory regions involved in the complex process that cause diseases [22]. Next-generation sequencing (NGS) provides rapid analyses of large quantities of genomic information, including DNA, mRNA, microRNA (miRNA), and noncoding RNA [23]. In the present study, we first reanalyzed the publicly available miRNA microarray dataset retrieved from GEO using NGS in combination with bioinformatic tools. A total of 52 DEGs were identified between the AF and SR groups, including 26 downregulated DEGs and 26 upregulated DEGs. Next, pathway enrichment analysis showed that these DEGs were primarily enriched in the pathological processes of immune response, energy metabolism, inflammation, apoptosis, and coagulation, while the changes in genetic material eventually led to electrical and structural remodeling in atrial tissue.

However, the genetic basis of AF pathogenesis is complex, involving modest contributions to disease risk from genetic variations in human genes. To further investigate the potential genetic pathological processes of AF and provide new noninvasive methods for the clinical diagnosis and treatment of this disease, the downregulated (CHRNA5, LOC150051, and PP12719) and upregulated (DHRS9, LOC101928304, and RYR1) hub genes were demonstrated to be involved in the regulation of multiple pathways and to have strong predictive power for the occurrence of AF. CHRNA5, located in 15q25.1, belongs to the superfamily of ligand-gated ion channels that mediate fast signal transmission at synapses, is typically expressed in the nervous system, and is involved in various functional processes, including cognition, learning, and memory [24]. Several studies have indicated that alterations in CHRNA5 expression and/or activity are significantly related to lung cancer associated with smoking [25, 26], as well as various neurological disorders, such as Alzheimer's disease (AD) [27], Parkinson's disease [28], and schizophrenia [26]. To the best of our knowledge, no investigation has observed an association between CHRNA5 and AF, and this report is the first to determine that the downregulation of CHRNA5 contributes to the pathophysiological mechanism of AF. DHRS9, also known as retinol dehydrogenase L (RDHL), has been identified as a member of the short-chain dehydrogenases/reductase (SDR) family that converts retinol to retinal. Previous studies indicated that the DHRS9 gene participates in the biological synthesis of all-transretinoic acid (atRA), which exhibits notable antitumor activity through inhibition of cell proliferation, induction of cell differentiation, and apoptosis and has been utilized in several cancer therapies [29, 30]. Therefore, we surmise that the upregulated gene DHRS9 could be involved in the structural remodeling of atrial myocardium in patients with AF by accelerating cell apoptosis and promoting cell differentiation. In addition, Riquelme et al. found that DHRS9 expression is a relatively specific and stable marker of *in vitro*-generated human macrophages [31]. It is well-known that increased macrophage accumulation occurs in the atrial tissue of patients with AF and exacerbates atrial electrophysiological remodeling, which could contribute to the expression of DHRS9. RYP1 is a member of a family of fungal proteins that includes Wor1, a master transcriptional regulator of the white-opaque transition required for mating in *Candida albicans*. Microarray analysis demonstrated that RYP1 is required for the expression of the vast majority of yeast-specific genes, including two genes that are linked to virulence [32]. However, further research on the relationship between RYP1 and diseases has not been reported to date. We first determined that the RPY1 gene is involved in the pathogenesis of AF and is positively related to five pathways (PANCREAS_BETA_CELLS, ESTROGEN_RESPONSE_LATE, CHOLESTEROL_HOMEOSTASIS, WNT_BETA_CATENIN_SIGNALING, and ESTROGEN_RESPONSE_EARLY) and negatively related to four pathways (HEDGEHOG_SIGNALING, APOPTOSIS, ALLORAFT_REJECTION, and OXIDATIVE_PHOSPHORYLATION). Currently, studies investigating the role of the remaining three DEGs (LOC150051, PP12719, and LOC101928304) have not been conducted; our future research will investigate these genes.

Recently, accumulating evidence has indicated that the immune-inflammatory response plays a crucial role in many cardiac pathophysiological processes, including ischemic cardiac injury and the postinfarction repair process, and this response is characterized by cytokine expression, immune regulation, neuroendocrine system activation, and intracellular signal transduction pathways. Hofmann et al. found that CD4+ T cells that became activated after MI played an important role in myocardial wound healing [33]. Wu et al. identified that CD8^+^ T cells in the AF group were significantly increased compared with those in the normal rhythm group and participated in the KRBOX1-AS1 and WEE1 network, which competed with endogenous factors and mediated myocardial tissue infiltration [22]. Nevertheless, our results suggested increased infiltration of APC_co_inhibition, Mast_cell, neutrophils, pDCs, T_cell_costimulation, and Th1_cells in atrial tissue of AF patients compared with the paired SR atrial tissue. Moreover, by analyzing the correlation between hub genes and immune cells, we observed that there were downregulated hub genes that were notably negatively correlated with the above-mentioned six kinds of immune cells. Therefore, we surmise that CHRNA5, LOC10150051, and PP12719 may reduce the involvement of APC_co_inhibition, Mast_cell, neutrophils, pDCs, T_cell_costimulation, and Th1_cells in the occurrence and maintenance of AF. However, regarding this possibility, further research is warranted to elucidate the complex interactions between the genes and immune cells.

The current study has several limitations. First, our data represent the second mining and analysis of previously published datasets, and the reliability of these results needs to be further supported by laboratory experiments and clinical trials. Second, the number of datasets was relatively small. However, taken together, these results indicate that the key genes identified in this study may serve as novel biomarkers and potential therapeutic targets for AF patients and may help to elucidate the molecular mechanisms underlying the pathology of AF.

## Figures and Tables

**Figure 1:** Flowchart diagram of the present study.

**Figure 2:** Two-dimensional PCA cluster diagram and heatmap and volcano plot of all DEGs. (a, b) Two-dimensional PCA cluster diagram before and after sample correction. (c) Heatmap of all DEGs. Red indicates relatively high expression, and green indicates relatively low expression. (d) The volcano plot of all DEGs; red represents upregulated DEGs, and green represents downregulated DEGs.

**Figure 3:** Pathway and process enrichment analysis. Heatmap of enriched terms related to the inputted list of DEGs, colored according to their *p* values (a). The correlation among the seven pathways (b).

**Figure 4:** Screening of the hub genes. (a) Misclassification error of the LASSO coefficient distribution. (b) Distribution of LASSO coefficients for 6 related genes and different colors represent different genes. (c) A Venn diagram was used to visualize the intersection of key markers obtained by the two algorithms. (d) BORUTA algorithm to screen key genes.

**Figure 5:** Expression levels of the six key genes in SR controls and AF patients in the validation set (GSE41177); *p* values < 0.05 were considered to be significant.

**Figure 6:** ROC curve of the diagnostic efficacy verification after respective fitting the six key genes to one variable.

**Figure 7:** Circos analysis of the relationships among six novel hub genes; red indicates a positive correlation, while green indicates a negative correlation.

**Figure 8:** GSVA results of genes involved in different signaling pathways in atrial tissue. Blue indicates a positive correlation, while green indicates a negative correlation.

**Figure 9:** Visualization of immune infiltration and correlation between the key genes and immune cells. (a) Violin plot visualizing the difference in immune infiltration between SR and AF; the SR group is marked in green, and the AF group is marked in yellow; *p* < 0.05 was considered statistically significant. (b) Correlation between the six hub genes and 29 types of immune cells; red indicates a positive correlation, while blue indicates a negative correlation; shading color and asterisks represent the value of the corresponding correlation coefficients.

## Data Availability

The data used to support the findings of this study are available from the corresponding author upon request.

## References

[1] Zhang Y. F., Meng L. B., Hao M. L., Yang J. F., Zou T. (2020). Identification of co-expressed genes between atrial fibrillation and stroke. *Frontiers in Neurology*.

[2] Lozano-Velasco E., Franco D., Aranega A., Daimi H. (2020). Genetics and epigenetics of atrial fibrillation. *International Journal of Molecular Sciences*.

[3] Panchal G., Mahmood M., Lip G. (2019). Revisiting the risks of incident atrial fibrillation: a narrative review. Part 1. *Kardiologia Polska*.

[4] Nguyen T. N., Hilmer S. N., Cumming R. G. (2013). Review of epidemiology and management of atrial fibrillation in developing countries. *International Journal of Cardiology*.

[5] van Ouwerkerk A. F., Hall A. W., Kadow Z. A. (2020). Epigenetic and transcriptional networks underlying atrial fibrillation. *Circulation Research*.

[6] Roselli C., Chaffin M. D., Weng L. C. (2018). Multi-ethnic genome-wide association study for atrial fibrillation. *Nature Genetics*.

[7] Gutierrez A., Chung M. K. (2016). Genomics of atrial fibrillation. *Current Cardiology Reports*.

[8] Kornej J., Husser D., Bollmann A., Lip G. Y. (2014). Rhythm outcomes after catheter ablation of atrial fibrillation. *Hämostaseologie*.

[9] Cai W., Li H., Zhang Y., Han G. (2020). Identification of key biomarkers and immune infiltration in the synovial tissue of osteoarthritis by bioinformatics analysis. *PeerJ*.

[10] Gautier L., Cope L., Bolstad B. M., Irizarry R. A. (2004). affy--analysis of Affymetrix GeneChip data at the probe level. *Bioinformatics*.

[11] Leek J. T., Johnson W. E., Parker H. S., Jaffe A. E., Storey J. D. (2012). The sva package for removing batch effects and other unwanted variation in high-throughput experiments. *Bioinformatics*.

[12] Leek J. T., Storey J. D. (2007). Capturing heterogeneity in gene expression studies by surrogate variable analysis. *PLOS Genetics*.

[13] Ritchie M. E., Phipson B., Wu D. (2015). Limma powers differential expression analyses for RNA-sequencing and microarray studies. *Nucleic Acids Research*.

[14] Diboun I., Wernisch L., Orengo C. A., Koltzenburg M. (2006). Microarray analysis after RNA amplification can detect pronounced differences in gene expression using limma. *BMC Genomics*.

[15] Hulsegge I., Kommadath A., Smits M. A. (2009). Globaltest and GOEAST: two different approaches for gene ontology analysis. *BMC Proceedings*.

[16] Ogata H., Goto S., Sato K., Fujibuchi W., Bono H., Kanehisa M. (1999). KEGG: Kyoto Encyclopedia of Genes and Genomes. *Nucleic Acids Research*.

[17] Friedman J., Hastie T., Tibshirani R. (2010). Regularization paths for generalized linear models via coordinate descent. *Journal of Statistical Software*.

[18] Robin X., Turck N., Hainard A. (2011). pROC: an open-source package for R and S+ to analyze and compare ROC curves. *BMC Bioinformatics*.

[19] Zeng H., Song X., Ji J., Chen L., Liao Q., Ma X. (2020). HPV infection related immune infiltration gene associated therapeutic strategy and clinical outcome in HNSCC. *BMC Cancer*.

[20] Zhou D., Chen Y., Wu J. (2019). Association between chymase gene polymorphisms and atrial fibrillation in Chinese Han population. *BMC Cardiovascular Disorders*.

[21] Ellinor P. T., Yoerger D. M., Ruskin J. N., Mac Rae C. A. (2005). Familial aggregation in lone atrial fibrillation. *Human Genetics*.

[22] Wu J., Deng H., Chen Q. (2020). Comprehensive analysis of differential immunocyte infiltration and potential ceRNA networks involved in the development of atrial fibrillation. *BioMed Research International*.

[23] van Dijk E. L., Auger H., Jaszczyszyn Y., Thermes C. (2014). Ten years of next-generation sequencing technology. *Trends in Genetics*.

[24] Zhan D., Yao Q., Fu S. (2019). Impact of CHRNA5 polymorphisms on the risk of schizophrenia in the Chinese Han population. *Molecular Genetics & Genomic Medicine*.

[25] le Marchand L., Derby K. S., Murphy S. E. (2008). Smokers with the CHRNA lung cancer-associated variants are exposed to higher levels of nicotine equivalents and a carcinogenic tobacco-specific nitrosamine. *Cancer Research*.

[26] Huang C. Y., Xun X. J., Wang A. J. (2015). CHRNA5 polymorphisms and risk of lung cancer in Chinese Han smokers. *American Journal of Cancer Research*.

[27] Dineley K. T., Westerman M., Bui D., Bell K., Ashe K. H., Sweatt J. D. (2001). Beta-amyloid activates the mitogen-activated protein kinase cascade via hippocampal alpha7 nicotinic acetylcholine receptors: in vitro and in vivo mechanisms related to Alzheimer's disease. *The Journal of Neuroscience*.

[28] Xie A., Gao J., Xu L., Meng D. (2014). Shared mechanisms of neurodegeneration in Alzheimer’s disease and Parkinson’s disease. *BioMed Research International*.

[29] Kropotova E. S., Zinovieva O. L., Zyryanova A. F. (2014). Altered expression of multiple genes involved in retinoic acid biosynthesis in human colorectal cancer. *Pathology and Oncology Research*.

[30] Hu L., Chen H. Y., Han T. (2016). Downregulation of DHRS9 expression in colorectal cancer tissues and its prognostic significance. *Tumor Biology*.

[31] Riquelme P., Amodio G., Macedo C. (2017). DHRS9 is a stable marker of human regulatory macrophages. *Transplantation*.

[32] Nguyen V. Q., Sil A. (2008). Temperature-induced switch to the pathogenic yeast form of Histoplasma capsulatum requires Ryp1, a conserved transcriptional regulator. *Proceedings of the National Academy of Sciences of the United States of America*.

[33] Hofmann U., Beyersdorf N., Weirather J. (2012). Activation of CD4+ T lymphocytes improves wound healing and survival after experimental myocardial infarction in mice. *Circulation*.

